# Visual Analysis of Research Hotspots in Geriatric Nursing Education in China and Abroad

**DOI:** 10.1155/2022/1796485

**Published:** 2022-04-18

**Authors:** Qingyun Li, Zihan Bu, Mengting Xue, Anle Huang, Wenjing Tu, Guihua Xu

**Affiliations:** Nanjing University of Chinese Medicine, Nanjing, China

## Abstract

**Background:**

This study aimed to conduct a literature search to determine research hotspots in the field of gerontological care education in China and abroad. A knowledge of the focus of research conducted abroad may assist Chinese educators in determining the shape of gerontological care education in the future.

**Methods:**

The “Web of Science Core Collection” and “CNKI” databases were searched for literature on gerontological care education published from 2010 to 2020. CiteSpace software was used to display the knowledge map of co-occurrence of keywords, and an evolution trend map of research hotspots in recent 10 years was constructed.

**Results:**

From 2010 to 2020, the focus of foreign gerontological nursing education research was on the training of gerontological nursing personnel; the development of elderly care services; and education and training in dealing with patients with senile delirium and dementia. The focus of gerontological nursing education research in China was primary care education, training of senior elderly nursing personnel, talent training mode reform, training of nursing staff, and career development paths for geriatric nursing staff.

**Conclusions:**

Foreign geriatric nursing education research focuses on cultivating talents, mental health services for the elderly, innovating the mode of pension, and the care of patients with disorders such as dementia and delirium, while in China, the emphasis remains on gerontological nursing personnel training. Attention to research developments in other countries may assist Chinese educators to promote the development of geriatric nursing education in our country.

## 1. Introduction

An aging society is defined as one in which members over 60 years old account for 10% of the total population, and those over 65 years old account for 7% of the total population [1]. China is currently in a fast-growing social model of population aging and aging population. According to the Forecast of Population Aging Trend in China: 2001–2100 Centenary, the first 20 years of the 21st century are a stage of rapid aging in this country. The number of elderly in China in 2020 is 248 million, and the aging level has reached 17.17% and is predicted to reach 400 million and more than 30% in 2050 [2]. While increases in the number of elderly call for new requirements in geriatric nursing education, its development in China appears to be lagging. How to develop geriatric nursing education and train professional nursing staff to meet the needs of the elderly and their medical and healthcare services is a problem requiring an urgent solution. Given this social background, we used CiteSpace II to conduct an in-depth exploration of the research status and development trends in domestic and foreign geriatric nursing education in the past 10 years, to provide an effective reference for the development of geriatric nursing education in China.

## 2. Methods

### 2.1. Data Sources

The “Web of Science Core Collection” and CNKI databases were used as retrieval sources. A Boolean logic operator was used to construct the retrieval expression, with the following formula: (I) the English search formula is TS=(”Geriatric Nursing” (Text word) AND “education” (Text word)), and the literature type is limited to article and review; (II) the Chinese search formula is as follows: search in CNKI: theme = “Nursing Education for the Elderly” and “Nursing for the Elderly” and “Nursing for the Elderly.” Fuzzy search, source journals for all journals. Year: January 1, 2010–present. Search results: 446 English and 687 Chinese sources (excluding 23 meetings and five newspapers).

### 2.2. Study Method

Bibliometrics was used to analyze the research hotspots in geriatric nursing education. This method involves the quantitative analysis of a discipline through mathematics and statistics. CiteSpace II is a visual analysis software tool used in bibliometrics and was developed at the School of Information Science and Technology of the University of Drexel in the United States [3].

### 2.3. Temporal Distribution of Literature

The time-domain changes in the number of documents can reflect the research enthusiasm of a discipline to some extent. This study compared the number of published articles on geriatric nursing education in China and abroad from 2010 to 2020, and a line chart (Figure 1) was drawn to facilitate researchers to intuitively observe the distribution of domestic and foreign geriatric nursing education literature.

### 2.4. Network Analysis of Keyword Co-Occurrence

Keywords are the extraction of the core content of the literature. Through the statistics and analysis of high-frequency keywords, research hotspots and important topics in a field can be determined [4]. CiteSpace II software counts the frequency of keywords based on word frequency analysis and displays it clearly in the form of visualization. This study used the software to produce the co-occurrence knowledge map of keywords in elderly care education and the evolution trend map of research hotspots over the past 10 years (Figure 2). At the same time, an in-depth analysis of the top 10 keywords (Table 1) shows the current research hotspots in China and abroad.

### 2.5. Research Frontier (Burst Detection)

CiteSpace II has a mutation detection function. Examining the changing trend of higher-frequency words, it can analyze the development trend and research direction of the subject field, which is helpful for researchers to predict scientific research trends and explore potential hotspots [5]. We used this software to make a comparison table of emergent words concerning elderly care education research at the frontiers of research in China and abroad (as shown in Table 2). Following each keyword in the table, there is an emergence bar, and each small cell of the bar represents a year. The red bar indicates the frequency of keyword searches in that year, and the length of the red cell represents the duration of the keyword emergence.

## 3. Results

### 3.1. Temporal Distribution of Literature

As shown in Figure 1, the domestic publication trend of articles can be roughly divided into two stages. In the first phase (from 2010 to 2012), the number of publications was decreasing. However, during the second phase (2012 to 2020), the number of articles published increased rapidly. Although there was a slight decline in 2012, 2016, and 2018, the number of articles published on aged care research reached its peak in 2017, with a total of 295 articles issued, and compared with 2010, the number of posts had increased nearly four times. In addition, the number of foreign publications is significantly higher than that in China, which shows that research on domestic aged care education started relatively late compared with foreign countries.

### 3.2. Research Hotspots

Figure 2 shows the time-axis knowledge graph. The analysis results of CiteSpace II software show there are 146 nodes and 492 connections in China and 221 nodes and 1,174 connections in foreign countries. In light of the top 10 keywords in Table 1, it can be concluded that foreign research hotspots on aged care are mainly concentrated in the following three areas: research on the cultivation of aged nursing personnel (education, attitude, knowledge, nurse); research related to the development of elder care services, advocating people-centered care (older adult, older people, care, geriatrics, people), and developing and innovating care models; and related disease education and training research, where the keywords are dementia and delirium. This suggests that when dealing with the problem of population aging in China, we should first focus on the research of elderly care-related theories, such as elderly care and nursing. Attention should be also paid to the cultivation of elderly nursing talents, such as nursing education, personnel training, elderly nursing specialties, nursing students, and nursing specialties. In addition, a focus on the exploration of career development paths for elderly nursing nurses should be explored. The results suggest the research focus in this country is on a nursing education model and talent training, and the nursing of elderly-related diseases has not yet been fully developed.

### 3.3. Research Frontiers

The frontiers of foreign geriatric nursing education are summarized as the following: (I) educational objects: the emergent words from 2010 to 2012 reveal the society's concern for nurses. From 2016 to the present, we have continuously put forward all-round research on nursing education. The country has made every effort to increase talent training to meet the ever-increasing demand for elderly care services and improve elderly care development. (II) Educational content and mode: the research on elderly care since 2010 has focused on psychological care, prevention, and rehabilitation, which has further promoted the improvement and development of nursing education models. (III) Evaluation of teaching results: the emerging words from 2011 to 2013 were validation, validity, randomized controlled trial, quality of life, and scale, indicating that more emphasis is placed on research on evaluation methods of teaching results, which will help improve the education system.

The frontiers of domestic geriatric nursing education can be divided into the following three stages: (I) the initial exploration and development stage: the emergent words from 2010 to 2013 mainly focus on the exploration of the theoretical basis and teaching methods of aged care, with the purpose of drawing on the relevant experience of foreign aged care to promote the development of disciplines. (II) The rapid development stage: from 2013 to 2018, with the rapid development of geriatric nursing education, the current situation of population aging has prompted a sharp increase in the demand for elderly nursing professionals. Various colleges and universities vigorously carry out the training of senior nursing professionals to provide talent reserves for the construction of the senior nursing service system. (III) Stability development stage: 2018 to the present is the stable development stage of China's elderly nursing education. This stage requires the training of elderly nursing talents at different levels according to social needs and further consolidates the construction of the professionalization of elderly nursing. However, the training of different types of elderly nursing talents in our country is still in the initial stage, and there is a need to continue to explore the core capabilities of various types of elderly nursing talents and improve the training system of elderly nurses with different levels of ability, as is practiced internationally.

## 4. Discussion

### 4.1. Foreign Research Hotspots

#### 4.1.1. Research on the Training of Elderly Nursing Talents

The training system for senior nursing talents abroad is relatively mature and adopts a hierarchical training model. For the training of junior talents, the research objects mainly include nursing students, in-service nurses, and undergraduates, and the content involves curriculum content, teaching methods, and attitudes to elderly cognitive practice. The American Association of Colleges of Nursing (AACN) schools released American Nursing Undergraduate Elderly Care Ability Standards and Curriculum Guidelines in 2010, clarifying 11 core competencies. Content on elderly care is included in the curriculum of nursing higher education, and requirements for elderly care nursing ability are inherent in the qualification examination content for registered nurses in the United States [6]. The WHO promulgated the Course Guide for Geriatric Nursing to clarify the continuing education goals of in-service nurses and further improve the professional skills of nurses in elderly care [7]. In terms of teaching methods, the teaching strategy of patient simulation is adopted [8], and narrative education and case studies are applied to the teaching of elderly nursing, focusing on practical experience, and fostering the willingness of nursing students to practice elderly nursing through good elderly nursing experience is highlighted [9]. Research on the training of senior elderly nursing talents abroad is not fully mature, and the research objects are mainly elderly nursing teachers, elderly masters, elderly doctoral students, and senior practice nurses. Based on evidence-based philosophy, the American Federation of Elderly Nursing Education has developed a wealth of elderly nursing programs and elderly nursing education courses, such as targeted training of elderly nursing teachers to address the shortage of teachers [10]. NEXUS, the American Federation of Nursing Education Exchanges, adopts distance teaching to offer senior nursing courses for nursing doctors [11]. The development of geriatric nursing is inseparable from the professional talents of geriatric nursing, and the specific methods of cultivating high-quality geriatric nursing talents are the focus of foreign research.

#### 4.1.2. Research on the Development of Elderly Care Services

The development of elderly care services and innovation in old-age care models are currently the research hotspot of foreign elderly care services. Facing the pressure of elderly care services, it is necessary to adopt a variety of elderly care models. The first of these calls for the adoption of environmental improvements, employee authorization, relationship reconstruction, and other methods to carry out cultural changes in nursing homes [12] to improve the quality of their services. Secondly, as public housing is the main place of residence that the elderly can afford, providing care for their life and spiritual needs can effectively reduce their burden on society by ensuring their ability to live independently. The third model calls for the promotion of the development of a village model of mutual assistance for the elderly to ensure consistency with family and community services. This measure can reduce the utilization rate of nursing homes and further reduce the burden on society. Finally, the case management method of long-term care should be adopted for the care of the elderly, and the care content and care plan are formulated through evaluation to reflect a people-centered care model [13]. The common development of multiple elderly care models is the first step to reduce the pressure on elderly care services. The fundamental solution is to strengthen the self-care ability of the elderly. Foreign countries have proposed the concept of productive aging, pointing out that the elderly can be paid through volunteer activities, production activities, or other unpaid activities to improve the value of their life and contribute to society [14] and achieve a successful model of aging. At the same time, research on the successful aging of the disabled elderly is also difficult in foreign research.

#### 4.1.3. Research on Disease Education and Training

At present, research on disease education and training abroad is mainly focused on the nursing care of patients with delirium and dementia. In this regard, foreign countries have proposed a human-centered care model, which is conducive to promoting agreement between patients and medical staff on treatment plans, thereby improving the quality of life of patients and reducing the burden on caregivers [15]. In this way, training on communication and education strategies for caregivers of dementia has become a top priority for the implementation of care work. Foreign countries currently adopt the MESSAGE plan [16], VIPS communication skill training [17], TANDEM communication plan [18], and other dementia care training programs to provide caregivers with structured and systematic communication skill training to improve their communication skills and quality of care. In addition, delirium can lead to the occurrence or aggravation of cognitive impairment in the elderly, resulting in damage to physical function and even death [19]. However, research abroad is in the preliminary stage of exploration in this regard and mainly focuses on the evaluation, prevention, and treatment of delirium. The education objects are mainly clinical nurses and family caregivers in the elderly care team, and the education places are mainly concentrated in hospitals, elderly care institutions, and families. The main forms of education are face-to-face education, distance education, and education manuals. van de Steeg et al. [20] carried out a three-month online learning training course for hospital clinical nurses, and the results showed that the course strengthened nurses' cognition of delirium in the elderly and increased its screening rate.

### 4.2. Domestic Research Hotspots

#### 4.2.1. Research on the Training of Elderly Nursing Talents

Promoting elderly nursing and developing specialist nurses are important tasks for the development of nursing during the 13th Five-Year Plan [21]. Research by related scholars pointed out that promoting the cultivation of aged nursing talents at different levels according to social needs is the current research focus of talent training [22]. Skilled, applied, and management-aged nursing talents should be cultivated to promote the sustainable development of the aged nursing profession in this country. Taylor's behavioral goal model theory supports [23] set training goals based on the core competence of nurses and, on the other hand, determining the content and methods of training based on the goals. It is easy to see that the construction of core competence is currently a research hotspot in the cultivation of elderly nursing talents. Scholars such as Li and Song [24] constructed the core competence system of elderly nursing for undergraduate nursing students, while Wang [25] constructed the core competence evaluation index of elderly care through qualitative research and continued to revise it [26]. In short, China is still in the exploratory stage of the training of senior nursing professionals and training high-quality senior nursing professionals should be a research focus for Chinese scholars.

#### 4.2.2. Research on the Reform of Talent Training Mode

Clinical nursing teaching methods are the focus of continuous attention in the reform of talent training models. At present, methods such as high-simulation nursing experimental teaching [27] and situational simulation teaching [28] are used in China. Set scenes with the support of information technology and the social needs of elder care encourage nursing students to actively participate in elder care and cultivate positive professional values to this care. Although the simulation teaching method has improved the effect of elderly nursing teaching, current research difficulties remain complicated, such as how to further enrich the material of simulation teaching, carry out interdisciplinary cooperation, and arrange the simulation plan reasonably. The content of talent training emphasizes the mode of combining quality education and innovation, takes nursing procedures and holistic nursing as supporting theories, cultivates dialectical thinking, and adds humanistic care courses. In addition, to meet the needs of elderly care services, the combination of medical care and nursing, school-enterprise joint training [29], school-hospital-community-nursing home training [30], and other training models is carried out. At present, the research hotspot of nursing talent training must match the positions and courses and train middle and high vocational senior nursing talents to increase the intensity of nursing talent training.

#### 4.2.3. Study on the Career Development Path of Elderly Nursing Nurses

The Several Opinions on Speeding up the Pension Service Business publication [31] formally put forward the model of a combination of medical care and pension, and the 13th Five-Year's notice of the development of the national cause of aging and pension system construction planning [21] also clearly requires that the health management rate of the elderly over 65 years old should reach more than 70%. Therefore, to optimize nursing resources, it is necessary to improve the utilization rate of related elderly nursing human resources. The National Nursing Development Plan (2016–2020) [32] and Guidance on Implementing Post Management of Hospital Nurses [33] pointed out that a clear nurse career development path is the basis of scientific management of nursing human resources, which explains why this development path is a current research hotspot.

### 4.3. Comparing the Research Hotspots at Home and Abroad

#### 4.3.1. Differences in Research Hotspots

Foreign countries focus on research related to elderly care services and disease education and training; domestic research focuses on the reform of talent training mode and career development path.

#### 4.3.2. Cause Analysis of Difference

In terms of talent training, the training of elderly nursing talents abroad is relatively mature, the training system of primary talents is relatively perfect, and the senior training is not yet fully mature; however, the training of senior professional nursing talents in China is still in the exploratory stage.

Therefore, the focus of domestic research lies in the basic fields such as talent training mode and career development path, while in foreign countries, due to their early start, the research focus tends to be more innovative fields such as elderly care services and disease education and training.

#### 4.3.3. Possible Results of Differences

Foreign prospective research will make some achievements in the successful aging and improving the quality of life of elderly patients and provide a rich experience in innovative models of elderly nursing. Due to the late start in China, the research will focus on cultivating high-quality elderly nursing professionals, reforming the talent training mode, and clarifying the career development path of elderly nurses combined with foreign experience. Therefore, in the future, a large number of professionals will emerge in the field of elderly care in China, forming a talent training model with competitiveness and development potential.

## 5. Conclusions

This study selects different databases, uses bibliometric methods to analyze the research hotspots of elderly nursing education, makes statistics on the results, and uses tools such as knowledge map and broken line map to realize visual display.

By comparing the research hotspots at home and abroad from the perspectives of differences, cause analysis, and result prospect, it can be found that the research hotspot of foreign geriatric nursing education has shifted from focusing on the training of elderly nursing talents, to research on innovative elderly service models, and finally to focusing on mental health services for the elderly. This series of changes is constantly improving and providing personalized care to promote a successful aging model. In view of the in-depth and extensive research on elderly nursing education, a relatively mature elderly nursing education and training system has been established abroad.

However, the current research hotspot in China is mainly focused on the training of elderly nursing personnel, and related elderly care services and dementia and delirium care services are still in the exploratory development stage. Therefore, carrying out research on nursing training for senile delirium and dementia is the top priority of current work. It is necessary to build a multidisciplinary nursing team education model that meets the characteristics of this country, promotes the management of related diseases, and improves the quality of elderly care services.

In summary, through the in-depth analysis of research hotspots in elderly nursing education in China and abroad, this article hopes to help domestic researchers grasp development trends, clarify future development directions and focus, and learn from foreign research results to further develop and improve related research on elderly nursing education, to promote the development of elderly nursing education in China.

## Figures and Tables

**Figure 1:** Number of publications on geriatric nursing education in China 2010–2020.

**Figure 2:** Knowledge map and research hotspot evolution trend map of keyword co-occurrence of geriatric nursing education in China and abroad from 2010 to 2020.

**Table 1:** Comparison of keywords of geriatric nursing education in China and abroad.

Serial	International		China	
	Keywords	Frequency	Keywords	Frequency
1	Education	91	Aged care	251
2	Care	74	Geriatric nursing	159
3	Older adult	57	Nursing	61
4	Attitude	55	Nursing education	43
5	Dementia	53	Talent development	40
6	Older people	44	Elderly care	38
7	Knowledge	43	Nurse	33
8	Geriatrics	42	Education	31
9	Nurse	41	Aging population	29
10	People	36	Nursing profession	28

**Table 2:** Comparison of research frontiers of geriatric nursing education in China and abroad from 2010 to 2020.

Serial	International		China	
	Emerging words	2010–2020	Emerging words	2010–2020
1	Nurse	■■□□□□□□□□□	Nursing	■■■□□□□□□□□
2	Depression	■■■■■□□□□□□	Geriatric nursing	■■■■□□□□□□□
3	Program	■■■□□□□□□□□	Education	■■□□□□□□□□□
4	Elderly people	□■■■■□□□□□□	Teaching	□■■■□□□□□□□
5	Geriatric nursing	□□■■■■□□□□□	Teaching method	□■■■■■□□□□□
6	Validation	□□□■■■■□□□□	Elderly care	□■■■■■□□□□□
7	Validity	□□□■■□□□□□□	Aging society	□□□□■■□□□□□
8	Prevention	□□□■■□□□□□□	Practical teaching	□□□□□■■■□□□
9	Rehabilitation	□□□□■■□□□□□	Higher vocational education	□□□□□□■■■□□
10	Randomized controlled trial	□□□□□■■□□□□□	Delphi	□□□□□□□□□■■
11	Quality of life	□□□□■■□□□□□	Nursing staff	□□□□□□□□□■■
12	Scale	□□□□■■□□□□□		
13	Perception	□□□□□■■□□□□		
14	Geriatric education	□□□□□■■□□□□		
15	Nursing student	□□□□□□□□■■■		
16	Frailty	□□□□□□□□■■■		

## Data Availability

The data used to support the findings of this study are available from the corresponding author upon request.
